The article "The Utilization of Chinese Herbal Products for Hyperthyroidism in National Health Insurance System (NHIRD) of Taiwan: A Population-Based Study" was published in 2022. Journal: Evid Based Complement Alternat Med.

# The Utilization of Chinese Herbal Products for Hyperthyroidism in National Health Insurance System (NHIRD) of Taiwan: A Population-Based Study

**DOI:** 10.1155/2022/5500604

**Published:** 2022-03-19

**Authors:** Cheng-Chieh Chang, Szu-Ying Wu, Yun-Ru Lai, Yu-Chiang Hung, Chung Y. Hsu, Hsuan-Ju Chen, Cheng-Chung Chu, Jai-Hong Cheng, Wen-Long Hu, Chun-En Aurea Kuo

**Affiliations:** ^1^Department of Chinese Medicine, Kaohsiung Chang Gung Memorial Hospital and Chang Gung University College of Medicine, No. 123, Dapi Rd., Niaosong Dist., Kaohsiung 833, Taiwan; ^2^School of Chinese Medicine for Post Baccalaureate I-Shou University, No.1, Sec. 1, Syuecheng Rd., Dashu District, Kaohsiung 84001, Taiwan; ^3^Department of Biological Science, National Sun Yat-Sen University, No. 70, Lien-hai Rd., Kaohsiung 80424, Taiwan; ^4^Department of Neurology, Chang Gung Memorial Hospital, Chang Gung University College of Medicine, No. 123, Dapi Rd., Niaosong Dist., Kaohsiung 833, Taiwan; ^5^Graduate Institute of Clinical Medical Science, College of Medicine, China Medical University, No. 91, Hsueh-Shih Rd., Taichung 40402, Taiwan; ^6^Management Office for Health Data, China Medical University Hospital, No. 2, Yuh-Der Rd., Taichung 40447, Taiwan; ^7^College of Medicine, China Medical University, No. 91, Hsueh-Shih Rd., Taichung 40402, Taiwan; ^8^Department of Computer Science, Tunghai University, No. 1727, Sec.4, Taiwan Boulevard, Xitun Dist., Taichung 407224, Taiwan; ^9^Center for Shockwave Medicine and Tissue Engineering, Kaohsiung Chang Gung Memorial Hospital, Chang Gung University College of Medicine, No. 123, Dapi Rd., Niaosong Dist., Kaohsiung 833, Taiwan; ^10^Medical Research, Kaohsiung Chang Gung Memorial Hospital, Chang Gung University College of Medicine, No. 123, Dapi Rd., Niaosong Dist., Kaohsiung 833, Taiwan; ^11^Kaohsiung Medical University College of Medicine, No. 100, Shihcyuan 1st Rd., Sanmin Dist., Kaohsiung 807, Taiwan; ^12^Fooyin University College of Nursing, No. 151, Chinhsueh Rd., Ta-liao Dist., Kaohsiung 831, Taiwan; ^13^Department of Leisure and Sports Management, Cheng Shiu University, No. 840, Chengcing Rd., Niaosong Dist., Kaohsiung 83347, Taiwan

## Abstract

**Background:**

Traditional Chinese Medicine (TCM) relieves associated symptoms of hyperthyroidism such as heat intolerance, palpitations, tremor, anxiety, weight loss, increased frequency of bowel movements, and shortness of breath. However, there are no studies regarding the core prescription patterns of herbal formula and single herbs for hyperthyroidism in Taiwan.

**Materials and Methods:**

This is a retrospective, observational study using the National Health Insurance Research Database (NHIRD) in Taiwan to analyze the prescription patterns of TCM. Demographic factors, such as sex, age, occupational status, and residential area, and the risk factors for hyperthyroidism were also studied.

**Results:**

The outpatient or/and inpatient services for hyperthyroidism receive 17,707 cases in a year. Overall, there were 13,394 newly diagnosed patients. TCM was used in 73% of the patients, and 77.3% of the patients were females. The acceptability of TCM was higher among female patients. Most patients were diagnosed with hyperthyroidism between the ages of 30 and 49 years. The most common comorbidity identified was diabetes mellitus. The most commonly prescribed Chinese herbal product (CHP) formula was Jia-Wei-Xia-Yao-San, while Xia-Ku-Cao was the most commonly prescribed single CHP. There was a high coprescription rate for Xuan-Shen, Bei-Mu, and Mu-Li.

**Conclusion:**

This study describes the core prescription pattern of TCM used in the treatment of patients with hyperthyroidism in Taiwan. The most frequently used CHPs could be potential candidates for future pharmacologic studies or clinical trials.

## 1. Introduction

Hyperthyroidism is a disease characterized by excessive levels of thyroid hormones in the blood. Thyroid hormones influence almost every tissue and organ system in the body. Graves' disease and toxic multinodular goiter are the two most common causes of hyperthyroidism [1]. The prevalence of hyperthyroidism is 0.75%, and its incidence rate is 51 per 100,000 per year in Europe [2]. Another report indicates that the prevalence of hyperthyroidism was 1.92% (2.95% in women and 0.94% in men), and its overall incidence was 96.1 per 100,000 during the observation period (2000–2008) in Taiwan [3]. The prevalence of hyperthyroidism increases with age. Hyperthyroidism is more frequent in women [1]. The clinical manifestations of hyperthyroidism include weight loss, osteoporosis, atrial fibrillation, embolic events, muscle weakness, tremor, neuropsychiatric symptoms, and rarely cardiovascular collapse and even death. It is essential to assess the severity of thyrotoxic manifestations, especially cardiovascular and neuromuscular complications, in order to formulate an appropriate treatment plan [4]. These features generally worsen without treatment. In fact, mortality due to these manifestations may reach 20%–50% before the introduction of satisfactory treatment [5]. Pregnant women, children, and the elderly are at increased risk for serious sequelae [6, 7].

The three main modalities used for the relief of symptoms and signs due to hyperthyroidism include medication, radioiodine, and thyroidectomy. Thionamides, propylthiouracil, and methimazole are the most commonly used antithyroid agents. Pruritus, urticaria, fever, arthralgia, and even abnormal taste are the common adverse effects of these drugs [8]. Radioactive iodine therapy is the most common form of therapy for Graves' disease. Moreover, it can also be used on toxic nodules and toxic multinodular goiter [9]. The major drawback of radioactive iodine is permanent hypothyroidism [10]. It is also contraindicated in pregnancy, breastfeeding, and in patients with severe ophthalmopathy. Surgical intervention such as thyroidectomy is usually accompanied by complications, including hypertrophic scarring, occipital headache, recurrent laryngeal nerve paralysis, hypocalcemia, and thyroid storm. This procedure has a mortality rate of 0.2% [11–13]. Studies regarding why patients with thyroid disease choose complementary and alternative medicine (CAM) list the following reasons: helping to cope with the side effects of medication and treatments including fatigue, dry mouth, weight gain, and mental “fogginess,” easing the stress and anxiety of medication and treatments, or worries about having a lifelong diagnosis, trying to help with their care or to treat or cure their disease [14]. In Taiwan, the most utilized CAM is traditional Chinese medicine (TCM). Therefore, many patients seek TCM for the combined treatment of hyperthyroidism in Taiwan.

TCM is an important component of healthcare in Taiwan and provides an alternative for hyperthyroidism treatment. Chinese herbal products (CHPs) represent the modern form of decoction, in powder form, with more consistent quality and convenience for patient use. The National Health Insurance (NHI) program fully reimburses patients for single or formula CHPs in Taiwan. Typically, TCM doctors prescribe CHPs with one or more herbal formulas combined with several single herbs based on the patient's symptoms. Traditional Chinese herbal medicines are mainly used in combination with antithyroid agents to treat hyperthyroidism. One systematic review suggested that traditional Chinese herbal medicines added to other routine treatments have therapeutic potential for people with hyperthyroidism, which may alleviate the symptoms and signs of hyperthyroidism, improve thyroid function, and reduce some adverse effects caused by antithyroid drugs, radioiodine, and thyroidectomy [15]. However, because of methodological limitations, the study was unable to provide strong evidence for the use of Chinese traditional herbal medicine in the treatment of hyperthyroidism or recommend any single preparation or formulation for clinical use. Therefore, the CHPs used for the treatment of hyperthyroidism and their prescription patterns are yet to be fully elucidated.

In Taiwan, the single-payer NHI program was launched on March 1, 1995. This NHI program provides 99% coverage for the inhabitants of Taiwan. The computerized reimbursement database of the NHI, the National Health Insurance Research Database (NHIRD), contains demographic data; dates of outpatient visits and hospitalizations; diagnostic codes based on the International Classification of Diseases, Ninth Revision, Clinical Modification (ICD-9-CM); and details of Chinese and Western medicine prescriptions. It can be used as a platform to understand the utilization of CHPs. Here, we aimed to evaluate the CHPs used for the treatment of hyperthyroidism and their prescription patterns in Taiwan. The epidemiology and comorbidities of hyperthyroidism in Taiwan were also investigated.

## 2. Materials and Methods

### 2.1. Data Sources

In this study, we used a subset of data from the NHIRD called the Longitudinal Health Insurance Database 2000 (LHID 2000). According to the NHI, there are no significant statistical differences in demographic factors (i.e., sex and age) between the LHID 2000 and the entire NHI database. Thus, the LHID 2000 may be representative of the characteristics of the general population of the whole nation. Before the release of the electronic files for research, personal identification numbers were encrypted to protect patient privacy. The study was approved by the Institutional Review Board of China Medical University and Hospital (CMUH104-REC2-115).

### 2.2. Study Population

The selection of study subjects from a random sample of one million individuals is presented in Figure 1. Of the one million randomly selected individuals in the LHID 2000, we identified 17,707 patients with newly diagnosed hyperthyroidism (ICD-9-CM 242.xx) between January 1, 1997, and December 31, 2013. To ensure the accuracy of the hyperthyroidism diagnosis, we selected patients who had more than three inpatient hospitalizations and/or western medical outpatient department visits. Patients diagnosed with hyperthyroidism before the end of 1999 (*n* = 3,448) and those who were younger than 20 years of age (*n* = 865) were excluded. In total, 13,394 patients with hyperthyroidism were included in the analysis. Patients with hyperthyroidism were then divided into two groups: those who visited TCM clinics for any indications at least once during the study period (TCM user) and those who never visited TCM clinics after the first hyperthyroidism diagnosis (TCM nonuser).

To determine the independent variables for the use of CHPs among patients with hyperthyroidism, we studied the demographic factors of sex, age, occupational status, and residential area and the risk factors for hyperthyroidism. Age was categorized into five ranges: 20–29, 30–39, 40–49, 50–59, and ≥60 years. Occupational status was categorized as one of the three classes: white-collar, blue-collar, and others. The survey of the population distribution in this study was based on the district branches of the National Health Insurance Administration, which consist of Northern Taiwan, Taipei, Central Taiwan, Southern Taiwan, Eastern Taiwan, and Kao-Ping (the most southern part of Taiwan).

### 2.3. TCM

The list of reimbursed CHPs was downloaded from the website of the Bureau of NHI. Corresponding drug information on a specific mixture or name was then obtained from the Committee on Chinese Medicine and Pharmacy website, including the proportions of each ingredient, date and period of drug approval, drug names, and manufacturers' codes.

## 3. Statistical Analysis

Differences in baseline characteristics between the TCM user and nonuser groups were examined using chi-squared tests and Fisher's exact tests for categorical variables and Student's *t*-tests for continuous variables. Multiple logistic regression was conducted to evaluate demographic characteristics (sex, age, occupational status, and residential areas) and comorbidities that correlated with TCM use. The model produced odds ratios (ORs) and corresponding 95% confidence intervals (CIs). Adjusted ORs were used to identify patients predicted to have higher odds of using TCM therapy. All statistical analyses were performed using SAS software version 9.4 (SAS Institute Inc., NC, USA). Two-tailed *p* values below 0.05 were considered significant.

## 4. Results

Among the one million randomly sampled patients from the NHIRD in 2000–2013, 17,707 patients received outpatient services more than 3 times and/or inpatient hospitalization claims for hyperthyroidism within one year. Excluding the patients diagnosed before 1999 and those younger than 20 years of age, there were 13,394 newly diagnosed patients. During the observation period, the overall incidence of hyperthyroidism was 83.6 per 100,000 per year in Taiwan. Among the above described patients, 9,822 received TCM treatment. Therefore, about 73% of the patients with hyperthyroidism used TCM treatment (Figure 1).

### 4.1. Demographic Characteristics

Female patients constituted 77.3% of the total patient population. More than 80% of the patients with hyperthyroidism receiving TCM treatment were women. Nearly half of the patients were diagnosed with hyperthyroidism at an age between 30 and 49 years. In addition, the patients who were between 20 and 49 years of age were more willing to receive TCM treatment. White-collar workers were much more susceptible to hyperthyroidism than blue-collar workers. Taipei, which is the capital of Taiwan, was the geographical area with the highest prevalence of hyperthyroidism. Diabetes mellitus was the most common comorbidity in patients with hyperthyroidism. The next most common comorbidities following diabetes mellitus were absence of menstruation, goiter, depression, osteoporosis, and asthma. Multivariable logistic regression was used to evaluate the effects of TCM on the risk of demographic characteristics and comorbidities, as indicated by the odds ratios (ORs) and 95% confidence intervals (CIs). The TCM treatment patients were significantly associated with a decreased risk of atrial fibrillation and congestive heart failure, in comparison with the non-TCM treatment patients. The TCM treatment patients were associated with a significantly higher risk of depression, asthma, and osteoporosis compared to the non-TCM treatment patients. Antithyroid drugs, which interfere with the synthesis of thyroid hormones, are the Western medication treatment of choice for thyrotoxicosis. The most common medication includes propylthiouracil (PTU), methimazole (MMI), and carbimazole (CMZ). The characteristics of Western medication use of TCM user and TCM nonuser are listed in Table 1.

### 4.2. Prescriptions for Hyperthyroidism

The most common TCM prescription pattern for patients with hyperthyroidism contained 5–8 combinations of a formula CHP or a single herb CHP. There was an average of 6.67 CHPs per single prescription (Figure 2). The three most commonly prescribed formula CHPs for hyperthyroidism were Jia-Wei-Xia-Yao-San (JWXYS), Zhi-Gan-Cao Tang, and Tian-Wang-Bu-Xin-Dan (Table 2). Xia-Ku-Cao (*Prunella vulgaris*) was the most commonly prescribed single CHP for patients with hyperthyroidism, followed by Dan-Shen (*Radix Salviae miltiorrhizae*), Xuan-Shen (*Scrophularia ningpoensis* Hemsl.), Bei-Mu (*Bulbus fritillariae cirrhosae*), and Mu-Li (oyster shell) (Table 2). The top five most commonly used combinations of two-formula CHPs were JWXYS/Zhi-Gan-Cao Tang, Zhi-Bo-Di-Huang-Wan/Zhen-Ren-Huo-Ming-Yin, Tian-Wang-Bu-Xin-Dan/JWXYS, Tian-Wang-Bu-Xin-Dan/Kan-Mai-Ta-Tsao-Tang, and JWXYS/San-Zhong-Kui-Jian-Tang (Table 3). Three of the five most commonly used combinations contain JWXYS. The top three most commonly prescribed two-single-CHP combinations were Xuan-Shen/Xia-Ku-Cao, Xuan-Shen/Bei-Mu, and Bei-Mu/Xia-Ku-Cao (Table 3).

## 5. Discussion

This is the first nationwide survey of hyperthyroidism in Taiwan using the NHIRD. There were 13,394 newly diagnosed patients among the one million randomly selected individuals. Over 73% of the hyperthyroidism patients received TCM treatment. TCM services are included in National Health Insurance coverage, and about 15% of medical institutions provide TCM services in Taiwan [16]. Moreover, the use of Chinese herbal products has been demonstrated to be effective against hyperthyroidism [15]. Because of the convenience, affordability, accessibility, and effectiveness of TCM services, over 70% of the hyperthyroidism patients utilize TCM services. The higher incidence of hyperthyroidism in this study may be due to the inclusion of both overt and subclinical hyperthyroidism [1].

Because the clinical manifestations of hyperthyroidism in the elderly are often atypical and can be attributed to other medical conditions, most patients diagnosed with hyperthyroidism are between 30 and 49 years of age [17, 18]. Also, based on previous studies, compared with the group aged <20 years, the group aged 35–49 years had the highest ratio of TCM users in 2000 and 2005 (AOR = 1.68; 1.61); the group aged 20–34 years had the highest ratio of TCM users in 2010 (AOR = 1.60) [19]. This can explain that the utilization of TCM treatment is more popular in hyperthyroidism patients aged 20–49 years. Hyperthyroidism occurs much more frequently in women than in men. This might be due to immune system differences, as women have been found to have a more intense genetic autoimmune background [20]. In one previous study, the ratio of TCM users in Taiwan among women was more than that among men in all 3 cohorts. This difference between genders in the number of TCM users increased gradually from 2000 to 2010 [19]. The trend is similar in our current study.

The relationship between emotional stress and the onset of hyperthyroidism has been well investigated [21]. More than 50% of the patients were white-collar workers. Taipei is the capital and economic center of Taiwan. The lifestyles of people in Taipei are more stressful than those of residents of other regions of Taiwan. In this LHID, approximately 40% of the patients with newly diagnosed hyperthyroidism were from Taipei. The utilization rate of TCM services is higher in the central part of Taiwan, which is consistent with the epidemiological characteristics in other NHIRD studies in Taiwan [16]. This may be attributable to the higher density of Chinese medicine physicians in this area. The most common comorbidity in patients with hyperthyroidism was diabetes mellitus. It has been reported that the incidence and prevalence of thyroid dysfunction are high among patients with type 1 and type 2 diabetes mellitus [22]. Menstrual disturbance is another frequent comorbidity in patients with hyperthyroidism. In addition, patients with severe hyperthyroidism have been shown to have a higher prevalence of secondary amenorrhea and hypomenorrhea [23]. This may be because high levels of circulating thyroid hormones augment the gonadotropin response [24]. In Taiwan, patients with amenorrhea are in favor of TCM treatment. TCM therapy has been shown to lead to holistic regulation of the reproductive system and can effectively treat gynecological diseases [25–27]. Depression is another common comorbidity that patients with hyperthyroidism are treated for using TCM. TCM is a popular option for the treatment of depression in oriental societies [28]. TCM may thus be beneficial for the treatment of mood-related illness including depression [29–31].

### 5.1. Commonly Used Formula CHPs for the Treatment of Hyperthyroidism

JWXYS was the most commonly prescribed formula CHP for the treatment of hyperthyroidism. JWXYS is a well-known and effective TCM for the treatment of liver qi stagnation and reinforcement of the spleen. It can remedy the common symptoms of hyperthyroidism, such as dyspnea, insomnia, palpitations, and dizziness [32, 33]. One previous study has reported that JWXYS can be used to treat patients with hyperthyroidism and maintain an euthyroid state without the use of antithyroid drugs [15].

Sinus tachycardia is the most common rhythm disturbance in patients with hyperthyroidism [34]. Between 5% and 15% of patients with hyperthyroidism present with atrial fibrillation [35]. In this survey, atrial fibrillation was presented in 1.8% of patients with hyperthyroidism. Zhi-Gan-Cao Tang is a TCM that has been used to alleviate palpitations. Modern pharmacological studies have also confirmed that Zhi-Gan-Cao Tang can inhibit arrhythmia (Table 4) [36–38]. In fact, Zhi-Gan-Cao Tang was the second most commonly prescribed formula CHP for the treatment of hyperthyroidism and the combination of JWXYS and Zhi-Gan-Cao Tang is the most commonly used two-formula CHP combination for the treatment of hyperthyroidism.

Tian-Wang-Bu-Xin-Dan has the promising effects on sleep disorder [39], which is the common symptom of hyperthyroidism. Zhi-Bo-Di-Huang-Wan combined with propylthiouracil can improve the hyperthyroidism patient's clinical symptoms, serum thyroid hormone levels, and serum antioxidant activity indexes [40]. Zhen-Ren-Huo-Ming-Yin ameliorates thymic enlargement in hyperthyroidism patients [41].

### 5.2. Commonly Used Single CHPs for the Treatment of Hyperthyroidism

The most commonly prescribed single CHP for patients with hyperthyroidism is Xia-Ku-Cao. According to TCM theory, Xia-Ku-Cao reduces swelling and resolves hard lumps [54]. In Waike Zhengzong (Orthodox Manual of External Diseases), which is a well-known historical TCM book regarding external medicine, goiters may be treated using Xia-Ku-Cao Tang, which contains Xia-Ku-Cao and Bei-Mu [55]. Modern studies have found that Xia-Ku-Cao has antioxidant, immunomodulatory, anti-inflammatory, and antitumor activity (Table 4) [42–44]. Dan-Shen is the second most commonly prescribed single CHP for patients with hyperthyroidism. It belongs to the Labiatae family and has been commonly used to “activate circulation and disperse stasis or sludging of blood in TCM practice.” Both alcohol and water extracts of Dan-Shen exhibit antioxidant, antiproliferative, and antiadipogenic effects [45]. This compound also has therapeutic effects in the treatment of Graves' orbitopathy (Table 4) [46, 47].

There is a high coprescription rate for Xuan-Shen, Bei-Mu, and Mu-Li. Xuan-Shen is shown to have anti-inflammatory, antiangiogenesis, and antioxidative activity (Table 4) [48–50]. The alkaloids from Bei-Mu have selective activity against muscarinic receptors and influence secretions from the thyroid gland (Table 4) [51]. Mu-Li is salty and astringent in flavor and is also indicated by TCM theory to soften hardness and dissipate nodules. It is mentioned in the Compendium of Materia Medica, which is one of the most famous medical books in the history of TCM, that Xia-Ku-Cao, Bei-Mu, and Mu-Li can be used to treat goiter. Medical Insights, which is an ancient practical traditional Chinese medicine book, indicates the use of the Chinese medical formula “Xiao-Luo-Pills” for the treatment of scrofula. Xiao-Luo-Pills are composed of Xuan-Shen, Bei-Mu, and Mu-Li. There are case reports demonstrating that Xiao-Luo-Pills can be used for the treatment of subacute thyroiditis and hyperthyroid heart disease (Table 4) [52, 53]. This may explain the high combination rate of Xuan-Shen, Bei-Mu, and Mu-Li.

### 5.3. Limitations

The NHI program only reimburses individuals for modern CHPs prescribed by TCM doctors. The usage of raw herbal medicine is thus not included in this survey. However, most patients with hyperthyroidism receiving TCM treatment still use modern CHPs due to the well-expanded coverage of NHI. Therefore, the impact of the above limitation on the results of this study may not be significant. Although we used some ways to focus on the populations of interest, we were unable to relate whether the subjects visited TCM for hyperthyroidism or other diseases, or whether they visited TCM for relieving symptoms of hyperthyroidism or the side effects of the medication. The findings of this study need to be carefully applied to clinical practice, and future study regarding each CHP in treating hyperthyroidism is warranted.

## 6. Conclusions

The acceptability of TCM was higher among female patients. A high percentage of patients with hyperthyroidism used TCM services in Taiwan. Diabetes mellitus was the most common comorbidity of hyperthyroidism. The most commonly prescribed formula CHP for hyperthyroidism was JWXYS. The most commonly prescribed single CHP was Xia-Ku-Cao. There was a high coprescription rate for Xuan-Shen, Bei-Mu, and Mu-Li.

This study draws some characteristics of TCM use in Taiwan. Understanding the prescription pattern used by TCM physicians, who usually prescribe according to TCM theories, this study may be useful for research on hyperthyroidism and its management. Therefore, the treatment mechanisms of frequently prescribed CHPs for hyperthyroidism, the safety issues, and drug-herb interactions should be prioritized in future research. The trend of TCM use discovered in this study could be applied for well-conducted, double-blind, randomized, placebo-controlled studies which aim to evaluate the efficacy of TCM on the management of hyperthyroidism.

## Figures and Tables

**Figure 1:** Flowchart describing the recruitment of subjects from LHID 2000 between 2000 and 2013 in Taiwan. TCM, traditional Chinese medicine.

**Figure 2:** Distribution of the number of CHPs per prescription. The most common TCM prescriptions for patients with hyperthyroidism contained 5–8 CHPs in a formula or a single CHP. There was an average of 6.67 CHPs per single prescription. CHP, Chinese herbal product; TCM, traditional Chinese medicine.

**Table 1:** Demographic characteristics and results of multiple logistic regression models. Adjusted odds ratios and 95% confidence intervals of patients with hyperthyroidism between 2000 and 2013 in Taiwan are shown.

Characteristics	TCM non-user *N* = 3572		TCM user *N* = 9822		*p* value	Adjusted^#^ OR (95% CI)	*p* value
	*n*	%	*n*	%			
No. of cases							
TCM for hyperthyroidism			416				
Sex					<0.001		
Women	2411	67.5	7944	80.9		1.00	
Men	1161	32.5	1878	19.1		0.52 (0.47–0.57)	<0.001
Age at diagnosis of hyperthyroidism, years					<0.001		
20–29	526	14.7	2070	21.1		1.00	
30–39	804	22.5	2579	26.3		0.83 (0.74–0.95)	0.005
40–49	799	22.4	2317	23.6		0.76 (0.67–0.86)	<0.001
50–59	681	19.1	1583	16.1		0.58 (0.51–0.67)	<0.001
≥60	762	21.3	1273	13.0		0.42 (0.37–0.49)	<0.001
Mean (SD)^†^	47.4	(16.0)	42.8	(14.1)	<0.001		
Occupational status					0.32		
White-collar	2009	56.2	5550	56.5		1.00	
Blue-collar	1260	35.3	3516	35.8		1.03 (0.94–1.12)	0.52
Others	303	8.48	756	7.70		0.95 (0.82–1.10)	0.52
Residential area					<0.001		
Northern	445	12.5	1102	11.2		1.00	
Taipei	1519	42.5	3821	38.9		1.03 (0.90–1.17)	0.70
Central	468	13.1	1928	19.6		1.68 (1.45–1.96)	<0.001
Southern	529	14.8	1316	13.4		1.01 (0.87–1.18)	0.86
Eastern	89	2.49	238	2.42		1.13 (0.86–1.49)	0.39
Kao-Ping	522	14.6	1417	14.4		1.09 (0.93–1.27)	0.29
Comorbidity							
Atrial fibrillation					<0.001		
No	3459	96.8	9697	98.7		1.00	
Yes	113	3.16	125	1.27		0.63 (0.48–0.83)	0.001
Congestive heart failure					<0.001		
No	3392	95.0	9543	97.2		1.00	
Yes	180	5.04	279	2.84		0.78 (0.63–0.96)	0.02
Goiter					0.12		
No	3330	93.2	9076	92.4		1.00	
Yes	242	6.77	746	7.60		1.03 (0.89–1.21)	0.67
Diabetes mellitus					<0.001		
No	3176	88.9	8977	91.4		1.00	
Yes	396	11.1	845	8.60		1.01 (0.88–1.15)	0.94
Pernicious anemia^‡^					0.61		
No	3570	99.9	9819	99.9		1.00	
Yes	2	0.06	3	0.03		0.70 (0.11–4.50)	0.71
Immune thrombocytopenia^‡^					0.54		
No	3567	99.9	9813	99.9		1.00	
Yes	5	0.14	9	0.09		0.68 (0.22–2.08)	0.50
Depression					<0.001		
No	3387	94.8	9117	92.8		1.00	
Yes	185	5.18	705	7.18		1.57 (1.32–1.86)	<0.001
Erectile dysfunction (only men)^§^					0.29		
No	1146	98.7	1843	98.1		1.00	
Yes	15	1.29	35	1.86		1.65 (0.86–3.15)	0.13
Absence of menstruation (only women)^&^					<0.001		
No	2243	93.0	7126	89.7		1.00	
Yes	168	6.97	818	10.3		1.19 (0.99–1.42)	0.06
Asthma					0.49		
No	3354	93.9	9188	95.6		1.00	
Yes	218	6.10	634	6.45		1.24 (1.05–1.47)	0.01
Intestinal malabsorption					0.99		
No	3570	99.9	9817	99.9		1.00	
Yes	2	0.06	5	0.05		0.68 (0.13–3.53)	0.64
Osteoporosis					0.85		
No	3336	93.4	9184	93.5		1.00	
Yes	236	6.61	638	6.50		1.21 (1.02–1.44)	0.03
Medication							
Carbimazole^#^	791	22.1	2189	22.3	0.86	0.97 (0.88, 1.07)	0.53
Methimazole^#^	1828	51.2	4518	46.0	<0.001	0.78 (0.71, 0.84)	<0.001
Propylthiouracil^#^	1123	31.4	3498	35.6	<0.001	1.12 (1.02, 1.22)	0.01

TCM, traditional Chinese medicine; OR, odds ratio; CI, confidence interval; SD, standard deviation. ^†^Student's *t*-test. ^‡^Fisher's exact test. ^#^Model adjusted for sex, age (categorical), occupational status, residential area, and comorbidity (except for erectile dysfunction and absence of menstruation). ^§^Model adjusted for age (categorical), occupational status, residential area, and comorbidity (except for absence of menstruation). ^&^Model adjusted for age (categorical), occupational status, residential area, and comorbidity (except for erectile dysfunction). ^*∗*^*p* < 0.05, ^*∗∗*^*p* < 0.01, and ^*∗∗∗*^*p* < 0.001.

**Table 2:** Top five formula CHPs and single CHPs prescribed by TCM physicians for the treatment of patients with hyperthyroidism between 2000 and 2013 in Taiwan (total prescriptions, *n* = 15,860).

Formula CHPs (number; frequency)	Number of person-days	Average daily dose (g)	Average duration for prescription (days)
Jia-Wei-Xia-Yao-San (533; 3.36%)	6411	4.9	12
Zhi-Gan-Cao Tang (400; 2.52%)	4396	4.1	11
Tian-Wang-Bu-Xin-Dan (327; 2.06%)	3090	4.8	9.4
Zhi-Bo-Di-Huang-Wan (151; 0.95%)	1357	4	9
Zhen-Ren-Huo-Ming-Yin (134; 0.84%)	1442	4	10.9

Single CHPs (number; frequency)			
Xia-Ku-Cao (420; 2.65%)	4486	3.1	10.7
Dan-Shen (319; 2.01%)	3390	1.2	10.6
Xuan-Shen (294; 1.85%)	2655	1.1	9
Bei-Mu (294; 1.85%)	3382	2.2	11.5
Mu-Li (273; 1.72%)	2738	1.2	10

TCM, traditional Chinese medicine; CHPs, Chinese herbal products.

**Table 3:** Top five most-used two-formula CHPs and two-single CHPs for the treatment of hyperthyroidism between 2000 and 2013 in Taiwan (total prescriptions, *n* = 15,860).

Two-formula CHPs	Number; frequency (%)	Number of person-days	Average daily dose (g)	Average duration for prescription (days)
Jia-Wei-Xia-Yao-San/Zhi-Gan-Cao Tang	106; 0.67	4396	4.9/4.1	11
Zhi-Bo-Di-Huang-Wan/Zhen-Ren-Huo-Ming-Yin	69; 0.44	1442	4/4	10.9
Tian-Wang-Bu-Xin-Dan/Jia-Wei-Xia-Yao-San	48; 0.3	3090	4.8/4.9	9.4
Tian-Wang-Bu-Xin-Dan/Kan-Mai-Ta-Tsao-Tang	48; 0.3	1367	4.8/3.8	11.7
Jia-Wei-Xia-Yao-San/San-Zhong-Kui-Jian-Tang	47; 0.3	1737	4.9/4.2	11.2

Two-single CHPs				
Xuan-Shen/Xia-Ku-Cao	140; 0.88	4486	1.1/3.1	10.7
Xuan-Shen/Bei-Mu	125; 0.79	2655	1.1/2.2	9
Bei-Mu/Xia-Ku-Cao	114; 0.72	3382	2.2/3.1	11.5
Xuan-Shen/Mu-Li	106; 0.67	2738	1.1/1.2	10
Mu-Li/Xia-Ku-Cao	93; 0.59	2338	1.2/3.1	11.6

CHPs, Chinese herbal products.

**Table 4:** Possible mechanisms of action or effects of frequently used CHPs for the treatment of hyperthyroidism.

Formula CHPs	Components	Mechanisms or effects
Jia-Wei-Xia-Yao-San	*Radix Bupleurum chinensis* *Rhizoma Atractylodis macrocephalae* *Radix Paeoniae alba* *Radix Angelica sinensis* *Radix Glycyrrhizae* *Poria cocos* *Radix Glycyrrhizae* *Radix Glycyrrhizae* *Herba Menthae* *Cortex Moutan* *Fructus Gardeniae* *Rhizoma Zingiberis Recens*	Sedative and antidepressive effects [32]; decreases the cardiovascular manifestations of hyperthyroidism [33]; maintains a euthyroid state in patients with hyperthyroidism [15]

Zhi-Gan-Cao Tang	*Panax ginseng* *Cinnamomum cassia Presl* *Zingiber officinale Rosc.* *Rehmannia glutinosa Libosch* *Ophiopogon japonicus (L.f.) Ker-Gawl.* *Cannabis sativa L.* *Colla corii asini* *Radix Glycyrrhiza*	Treatment for premature ventricular contractions [36]; prolongs field action potential duration in patients with atrial fibrillation [37]; decreases supraventricular arrhythmia and premature ventricular contraction [38]

Tian-Wang-Bu-Xin-Dan	*Rehmannia glutinosa* *Angelica sinensis* *Schisandra chinensis* *Ziziphus zizyphus* *Platycladus orientalis* *Asparagus cochinchinensis* *Ophiopogon japonicus* *Scrophularia ningpoensis* *Polygala tenuifolia* *Salvia miltiorrhiza* *Codonopsis pilosula* *Poria coco* *Platycodon grandiflorum*	Improving insomnia [39]

Zhi-Bo-Di-Huang-Wan	*Anemarrhena asphodeloides* *Phellodendron amurense* *Rehmannia glutinosa* *Cornus officinalis* *Dioscorea polystachya* *Alisma plantago-aquatica* *Poria cocos* *Cortex Moutan Radicis*	Improving clinical symptoms, serum thyroid hormone levels, and serum antioxidant activity indexes in hyperthyroidism [40]

Zhen-Ren-Huo-Ming-Yin	*Lonicerae japonicae flos* *Citri Reticulatae Pericarpium* *Angelicae sinensis Radix* *Saposhnikoviae Radix* *Angelicae dahuricae Radix* *Glycyrrhizae Radix et Rhizoma* *Fritillariae ussuriensis bulbus* *Trichosanthis Radix* *Olibanum* *Myrrha* *Gleditsiae Spina*	Ameliorating thymic enlargement in hyperthyroidism [41]

Single CHPs		

Xia-Ku-Cao	*Prunella vulgaris*	Reduces swelling and resolves hard lumps; possesses antitumor and possible immunomodulation effects [42]; possesses anti-inflammatory effects and is used to treat diseases due to excessive activation of the complement system [43, 44]

Dan-Shen	*Radix Salviae miltiorrhizae*	Exhibits antioxidant, antiproliferative, and antiadipogenic effects [45]; used to treat Graves' orbitopathy [46, 47]

Xuan-Shen	*Scrophularia ningpoensis Hemsl.*	Possesses potent antioxidative activity [48] and antiangiogenic activity [49, 50]

Bei-Mu	*Bulbus Fritillariae cirrhosae*	Possesses selective activity against muscarinic receptors and influences secretions from the thyroid gland [51]

Mu-Li	Oyster shell	Softens hardness and dissipates nodules according to TCM theory; treatment for subacute thyroiditis and hyperthyroid heart disease [52, 53]

## Data Availability

The dataset of this study is available from the NHIRD provided by the Bureau of National Health Insurance, Department of Health, and managed by the National Health Research Institutes. However, these data were used under policies limited only for the current study. Thus, the data are not publicly available.
